RETRACTED

# Alteration of astrocytes and Wnt/β-catenin signaling in the frontal cortex of autistic subjects

**DOI:** 10.1186/1742-2094-9-223

**Published:** 2012-09-21

**Authors:** Fujiang Cao, Ailan Yin, Guang Wen, Ashfaq M Sheikh, Zujaja Tauqeer, Mazhar Malik, Amenah Nagori, Michael Schirripa, Frank Schirripa, George Merz, Shiqing Feng, W Ted Brown, Xiaohong Li

**Affiliations:** 1 Department of Neurochemistry, NY State Institute for Basic Research in Developmental Disabilities, 1050 Forest Hill Road, Staten Island New York, USA; 2 Department of Developmental Neurobiology, NY State Institute for Basic Research in Developmental Disabilities, 10314, New York, NY, USA; 3 Digital Microscopy, NY State Institute for Basic Research in Developmental Disabilities, 10314, New York, NY, USA; 4 Department of Orthopaedics, General Hospital of Tianjin Medical Universtiy, Tianjin, China

**Keywords:** Autism, Astrocytes, Morphology, Wnt/β-catenin pathway, Neural plasticity

## Abstract

**Background:**

Autism is a neurodevelopmental disorder characterized by impairments in social interaction, verbal communication and repetitive behaviors. To date the etiology of this disorder is poorly understood. Studies suggest that astrocytes play critical roles in neural plasticity by detecting neuronal activity and modulating neuronal networks. Recently, a number of studies suggested that an abnormal function of glia/astrocytes may be involved in the development of autism. However, there is yet no direct evidence showing how astrocytes develop in the brain of autistic individuals.

**Methods:**

Study subjects include brain tissue from autistic subjects, BTBR T + *tf*J (BTBR) and Neuroligin (*NL*)-3 knock-down mice. Western blot analysis, Immunohistochemistry and confocal microscopy studies have been used to examine the density and morphology of astrocytes, as well as Wnt and β-catenin protein expression.

**Results:**

In this study, we demonstrate that the astrocytes in autisitc subjects exhibit significantly reduced branching processes, total branching length and cell body sizes. We also detected an astrocytosis in the frontal cortex of autistic subjects. In addition, we found that the astrocytes in the brain of an *NL3* knockdown mouse exhibited similar alterations to what we found in the autistic brain. Furthermore, we detected that both Wnt and β-catenin proteins are decreased in the frontal cortex of autistic subjects. Wnt/β-catenin pathway has been suggested to be involved in the regulation of astrocyte development.

**Conclusions:**

Our findings imply that defects in astrocytes could impair neuronal plasticity and partially contribute to the development of autistic-like behaviors in both humans and mice. The alteration of Wnt/β-catenin pathway in the brain of autistic subjects may contribute to the changes of astrocytes.

RETRACTED

## Background

Autism is a neurodevelopmental disorder characterized by impairments in social interaction, verbal communication and repetitive behaviors. But the etiology of this disorder is poorly understood. Animal models offer opportunities for conducting biological studies to understand the mechanisms responsible for the phenotypes. The BTBR T + *tf*J (BTBR) mice are currently used as a mouse model for understanding mechanisms that may be responsible for the pathogenesis of autism since they demonstrate the three core autistic symptoms [1-4]. In addition, the Neuroligin-3(*NL3*) knockdown mouse may be a useful model for studying autistic-related behaviors since this mouse model mimics autistic core symptoms [5].

The brain consists of two major cell types - neurons and glial cells. In the past, neurons have been extensively studied. However, research on glial cells has increased in the last decade. The development of the nervous system requires choreographed neuronal migration, axon guidance, target selection, dendritic growth and synapse formation.

Proper orchestration of each of these stages of neuronal development requires glial-derived factors. Glial cells in the central neural system (CNS) are categorized into four types, which include astrocytes, oligodendrocytes, microglia, and chondroitin sulfate proteoglycan *NG2*-positive cells. Astrocytes are a very heterogeneous population of cells, which interact with neurons and blood vessels. These cells detect neuronal activity and can modulate neuronal networks. Oligodendrocytes (or Schwann cells in the peripheral nervous system) form myelin and thus are prerequisites for the high conduction velocity of axons in vertebrates. Microglia cells are the immune cells of the CNS and respond to changes in the environment [6]. Together these cells play essential roles in nervous system development and function, from simple trophic support of neurons, and wrapping axons and allowing for rapid nerve impulse conduction, to modulating synaptic connectivity and efficacy. During nervous system development, the neural progenitor cells (NPCs) generate neurons first, followed by glia. The switch from neuron to glia at the proper time is critical for the establishment of normal brain function. The mechanisms regulating this transition and development of glia are complex, and currently are poorly understood [7]. However, a number of recent studies indicate that the fate switch is governed by both extrinsic environmental cues that promote astrogenesis in NPCs and NPC-intrinsic mechanisms that decrease neurogenic and increase astrogenic competence over developmental time. The Wnt(wingless-type MMTV integration site1) pathway has been shown to be required for the activation of the proneural genes neurogenin1 (*ngn1*) and neurogenin2 (*ngn2*) in NPCs, where, at an early stage, they act to promote neuronal differentiation [8-10]. Recently, Episcopo *et al*. demonstrated that Wnt1-regulated Frizzled-1/β-Catenin signaling pathway can also act as a candidate regulatory circuit controlling mesencephalic dopaminergic neuron-astrocyte crosstalk [11]. In addition, it was shown that Wnt**/**β-Catenin signaling increases in proliferating NG2+ progenitors and astrocytes during post-traumatic gliogenesis in the adult brain [12].

RETRACTED

Recently, a number of studies have suggested that abnormal functioning of glia/astrocytes may play a role in the development of autism. Laurence and Fatemi reported that the glial fibrillary acidic protein (GFAP), a marker for astrocytes, is elevated in the superior frontal, parietal and cerebellar cortices of autistic subjects [13]. GFAP was also reported to be three times higher in the cerebrospinal fluid of autistic and autistic-like conditions as compared with a control group [14]. In addition, a study reported that the expression of the astrocytic markers aquaporin4 and connexin43 are altered in the brains of subjects with autism. Most recently, a role for glia in the progression of Rett syndrome (RTT), an X-linked autism spectrum disorder caused by loss of function of the transcription factor methyl-CpG-binding protein 2 (*MeCP2*), has been reported [15-17]. In these studies, it was found that mutant astrocytes from an RTT mouse model and their conditioned medium, fail to support normal dendritic morphology of either wild-type or mutant hippocampal neurons. It was also shown that in globally *MeCP2*-deficient mice, re-expression of *Mecp2* preferentially in astrocytes significantly improved locomotion and anxiety levels, restored respiratory abnormalities to a normal pattern, and greatly prolonged lifespan compared to globally null mice. Furthermore, a recent study demonstrated that astrocytes in the fragile × mouse model induced developmental delays in normal dendrites including maturation and synaptic protein expression, and implicated a role for astrocytes in the development of the fragile × syndrome [18]. Taken together, the evidence suggests that glia/astrocytes could develop or be regulated abnormally in the autistic brain and that alterations of glia/astrocytes could be critically involved in the pathogenesis of autism. However, as yet there is no study directly investigating how astrocytes develop in the brain of autistic individuals. The aim of this study was to examine the development and morphology of astrocytes in the brains of autistic subjects, as well as in the brains of BTBR mice and *NL3* knockout murine models of autism.

RETRACTED

## Methods

### Study subjects

Frozen human brain tissues of six autistic subjects (mean age ± SD, 8.3 ± 3.8 years) and six age-matched normal subjects (mean age 8.0 ± 3.7 years) were obtained from the NICHD Brain and Tissue Bank for Developmental Disorders. Donors with autism fit the diagnostic criteria of the Diagnostic and Statistical Manual-IV, as confirmed by the Autism Diagnostic Interview-Revised. Participants were excluded from the study if they had a diagnosis of fragile × syndrome, epileptic seizures, obsessive-compulsive disorder, affective disorders, or any additional psychiatric or neurological diagnoses. This study was approved by the Institutional Review Board of the NY State Institute for Basic Research and the subjects’ information is summarized in Table 1.

**Table 1:** Study subject information

**Case**	**Age**	**Sex**	**Group**	**PMI(h)**	**Seizure**	**Retardation**	**Medication**	**Cause of death**
1	7	M	Control	12	-	-	Concerta, Clonidone	Drowning
2	8	M	Control	36	-	-	-	Drowning
3	4	F	Control	21	-	-	-	Lymphocytic myocarditis
4	9	F	Control	20	-	-	Albuterol, Zirtec	Asthma
5	6	M	Control	18	-	-	-	Multiple injuries
6	14	M	Control	16	-	-	-	Cardiac arrhythmia
7	7	M	Autism	20	-	-	-	Drowning
8	8	M	Autism	16	-	-	-	Drowning
9	4	F	Autism	13	-	-	-	Multiple injuries
10	9	F	Autism	24	-	-	-	Smoke inhalation
11	8	M	Autism	12	-	+	-	Drowning
12	14	M	Autism	12	+	+	-	Drowning

M, male; F, female; PMI (h) (Post-Mortem Intex).

Six BTBR *T + tfJ* (BTBR) mice and six age- and sex-matched B6 mice (7 weeks old) were obtained from the Jackson Laboratories (Bar Harbor, ME, USA). Mice were housed for 24 hours with food and water *ad libitum*to ease the stress before sacrifice. Then the mice were rapidly sacrificed with cervical dislocation for removal of the brains. All procedures were conducted in compliance with the NIH Guidelines for the Care and Use of Laboratory Animals and approved by the New York State Institute for Basic Research Institutional Animal Care and Use Committee.

The NL3 mouse was obtained by microinjection of neuroligin 3 RNAi into the fertilized CD-1 mouse and then transferring to the oviduct of surrogate CD-1 female mice. PCR analysis was conducted to confirm that it was a positive *NL3* knockdown founder mouse. A number of behavioral tests including open field test, elevated plus maze, water maze, vocalization test and social behavior test were carried out to determine the mouse behavior. The *NL3* mouse exhibited increased anxiety, impaired cognition, vocal communication deficits and decreased social interaction, compared with the age- and sex-matched littermate control mice (unpublished data).

RETRACTED

### Preparation of brain homogenates

The frontal cortex and cerebellum were dissected. The frozen frontal cortex and cerebellum tissues were homogenized (10% w/v) in cold buffer containing 50 mMTris–HCl (pH 7.4), 8.5% sucrose, 2 mM EDTA, 10 mM β-mercaptoethanol and a protease inhibitor cocktail (Sigma-Aldrich St. Louis, MO USA). The protein concentrations were assayed by the Bradford method [19].

### Immunohistochemistry

Paraffin sections (6 μm)were deparaffinized with xylene (2×), ethanol of 100% (2×), 80%, 50%, and 25% concentration and washed in TBS, 5 minutes each time. The sections were then incubated with primary antibodies overnight at 4°C. After washing in TBS for 5 minutes, the sections were further incubated with secondary antibody (biotinylated horse anti-mouse IgG, or biotinylated horse anti-rabbit IgG, VectaStain Elite ABC Kit, Vector Lab Burlingame, CA, USA) for 30 minutes at room temperature, followed by incubation in Avidin-biotinylated peroxidase (VectaStain Elite ABC Kit) for 45 minutes at room temperature and in 0.0125 g DAB/25 ml 0.05 M TBS/1 drop 30% H_2_O_2_ for 10 minutes at room temperature. All sections were washed in sequence with TBS, 25%, 50%, 80%, and 100% ethanol (2×) and xylene (2X) before mounting for viewing under the microscope.

### Western blot analysis

Brain homogenate samples in SDS sample buffer (20% glycerol, 100 mMTris, pH 6.8, 0.05% Bromophenol blue (w/v), 2.5% SDS (w/v), 250 mM DTT) were denatured by heating at 100°C for 5 minutes. Twenty to sixty micrograms of protein per lane per subject were loaded onto a 10% acryl-bisacrylamide gel and electrophoresed for 2 hours at 110 V at room temperature. The separated proteins were electroblotted onto a polyvinylidenedifluoridePVDF membrane for 1 hour at 100 V at room temperature. Protein blots were then blocked with 5% non-fat milk in PBS with 0.1% Tween-20 (PBST). After blocking, the blots were incubated with primary antibody overnight at 4°C followed by secondary antibody incubation for 1 hour at room temperature (goat ant-mouse IgG or goat anti-rabbit IgG, horse radish peroxidase (HRP)-conjugated, 1:5000, Sigma). After three washes in PBST (10 minutes each time), the blots were exposed to Hyper film ECL. Sample densities were analyzed with Image J software (NIH), an open domain Java image processing system. The densities of the protein expression bands, as well as the β-actin expression bands were quantified with background subtraction.

### Confocal microscopy and data analysis

Immunostaining images were visualized using a laserscanning confocal microscope to obtain clear pictures (Nikon Eclipse 90I, 10 × 40 maglification, IBR-Microscopy Shared Research Facility). Image J analysis was used to calculate area and immunostaining density. Quantification of western blot analysis was performed by Image J analysis and the internal standard beta-actin was used throughout.

RETRACTED

### Statistical analysis

Statistical analysis was conducted using SPSS 13.0 software. Means, standard deviations and standard errors of the mean were determined in sets of study subjects versus control subjects. The unpaired *t*-test was used to compare each parameter measured and *P* values were determined. *P* < 0.05 was considered statistically significant.

## Results

### The density and morphology of astrocytes were significantly changed in the frontal cortex of autistic subjects

With immunohistochemistry studies using anti-GFAP antibody, and employing confocal microscopy, we observed that the number of astrocytes was clearly increased. Quantitative analysis conducted on the brain slices from six autistic subjects and six age-matched normal controls showed that the density of astrocytes was increased approximately 1.6-fold in the frontal cortex of autistic subjects compared with age-matched controls (*P* = 0.035, Figure 1A). We also observed that the astrocyte morphology was grossly changed in the autistic cortex. With Image J analysis, we showed that the number of astrocytic branch processes radiating from the cell body was significantly decreased by 60.2% in the autistic subjects compared with the controls (*P* = 0.027, Figure 1A). The total branching length was significantly decreased by 71% compared with the controls (*P* = 0.007, Figure 1A). We examined cell body sizes and found that the mean cell body size of the autistic subjects was decreased by 37% compared to controls (*P* = 0.0001, Figure 1A). We examined cerebellar astrocytes of both autistic and control subjects. Our results demonstrated that their density and morphology were not significantly different in the autistic cerebellum compared with the controls (*P* = 0.088 for density of astrocytes; *P* = 0.065 for branch processes; *P* = 0.349 for total branch length and *P* = 0.124 for cell body size, Figure 1B).

**Figure 1:** **The morphology and density of astrocytes were significantly changed in the frontal cortex of autistic subjects.** Immunohistochemistry studies were carried out on frontal cortex (**A**) and cerebellum sections (**B**) from six autistic subjects and six age-matched controls using an anti-glial fibrillary acidic protein (GFAP) antibody (dilution 1:1000). Pictures were taken under both low power (LP) and high power (HP). Immunostaining of GFAP (dark brown color) was present in all astrocytes. The density of astrocytes, number of astrocytic branch processes, cell body size and the total branch length were quantified using Image J analysis. *P < 0.05, ***P < 0.001. Scale bar: 20 μm. Data are shown as mean ± standard error (SE).

RETRACTED

### The density and morphology of astrocytes in the brain of BTBR mice

Since BTBR mice exhibit autistic-like behaviors and are currently used as a mouse model to study autism, we examined whether their astrocytes have similar changes. Our results analyzed from six BTBR mice and six age-matched B6 mice showed that the density of astrocytes in the brain of BTBR mice was not significantly changed compared with control B6 mice(*P* = 0.069, Figure 2). In addition, we also examined the morphology of astrocytes in both BTBR and control B6 mice. With Image J analysis, we showed that the number of astrocytic branch processes in BTBR mice was not significantly different compared with B6 mice (*P* = 0.11, Figure 2). Both the total branching length and cell body size also remained unchanged in BTBR mice compared with the B6 mice (*P* = 0.178 and *P* = 0.431 respectively, Figure 2). These results suggest that both the density and morphology of astrocytes in BTBR mice are not significantly altered compared with B6 mice.

**Figure 2:** **The density and morphology of astrocytes in the brain of BTBR mice.** Immunohistochemistry studies were carried out on whole brain sections from six BTBR mice and six age-matched control B6 mice using an anti-glial fibrillary acidic protein (GFAP) antibody (dilution 1:1000). Immunostaining of GFAP (dark brown color) was present in all astrocytes. The density of astrocytes, number of astrocytic branch processes, cell body size and the total branch length were quantified using Image J analysis. Scale bar: 5 μm. Data are shown as mean ± standard error (SE).

To further confirm the results, we examined the GFAP expression level in the brain of BTBR and B6 mice with western blot analyses. Our results demonstrated that there are no significant differences in the GFAP expression between the frontal cortex (*P* = 0.12), as well as the cerebellum (*P* = 0.36) of BTBR and B6 mice (Figure 3).

**Figure 3:** **GFAP protein expression in the frontal cortex of BTBR and B6 mice.** Western blot analyses were carried out on frontal cortex and cerebellum homogenates from six BTBR mice and six age-matched B6 mice using anti-glial fibrillary acidic protein (GFAP) antibody (dilution 1:1000). The blots on cortex and cerebellum were quantified respectively after being normalized by actin (lower left bar figure for cortex and lower right bar figure for cerebellum). Data are shown as mean ± standard error (SE).

RETRACTED

### The morphology of astrocytes was altered in the brain of a NL3 knockdown mouse

In this study, we only obtained one *NL3* knockdown B6 mouse. These mice exhibit autism-like behaviors including increased anxiety, impaired cognition, vocal communication deficits and decreased social interactions. We found that the astrocytes in the frontal cortex of the *NL3* knockdown mouse exhibited similar changes to those that we observed in the frontal cortex of autistic subjects. We found that the number of astrocytic branch processes was decreased by 41.3% in the *NL3* knockdown mouse compared with the control B6 mouse (*P* = 0.01, Figure 4). The total branching length was also decreased by 52.6% compared with the control B6 mice (*P* = 0.022, Figure 4). In addition, we found that the mean value of the cell body size in the NL3 knockdown mouse was decreased by 43.7% compared with the control B6 mouse (*P* = 0.020, Figure 4). However, the density of astrocytes in the *NL3* knockdown mouse was not significantly changed compared with the control B6 mouse (*P* = 0.11, Figure 4).

**Figure 4:** **The morphology of astrocytes was altered in the frontal cortex of NL3 knockdown mice.** Immunohistochemistry studies were carried out on the whole brain sections from one NL3 knockdown mouse and one age-matched control littermate using an anti-glial fibrillary acidic protein (GFAP) antibody (dilution 1:1000). Immunostaining of GFAP (dark brown color) was present in all astrocytes. The density of astrocytes from the frontal cortex, as well as the number of astrocytic branch processes, cell body size and the total branch length were quantified using Image J analysis. *P < 0.05. Scale bar: 10 μm. Data are shown as mean ± standard error (SE).

### Wnt/β-catenin pathway signaling may be impaired in the brain of autistic subjects

Since the Wnt/β-catenin pathway has been suggested to play a role in controlling mesencephalic dopaminergic neuron-astrocyte crosstalk and is involved in the modulation of gliogenesis, we examined how the Wnt/β-catenin pathway is regulated in the autistic brain. By immunohistochemistry studies using anti-Wnt antibodies, we observed by confocal microscopy that the immunostaining was weaker in the neuronal cells of the frontal cortex of autistic subjects compared with the controls. Quantitative analysis showed that the immunoreactivity of Wnt was decreased in the autistic brain by 61% compared with the controls (*P* = 0.037, Figure 5). In addition, western blot studies were conducted to examine β-catenin protein expression in the brain of autistic subjects. Our results demonstrated that the mean value of β-catenin protein expression was decreased by 24.7% in the frontal cortex of autistic subjects (*P* = 0.002, Figure 5), but was not significantly changed in the autistic cerebellum compared with controls (data not shown). These results suggest that Wnt/β-catenin signaling activities may be down-regulated in the frontal cortex of autistic subjects.

RETRACTED

**Figure 5:** **Wnt and β-catenin protein expression in the brain of autistic subjects.** Upper panel: western blot analyses were carried out on frontal cortex homogenates from six autistic subjects and six age- and sex-matched controls using an anti-β-catenin antibody (dilution 1:1000) (5**A**). The blots were quantified after being normalized by actin (5**B**). Data are shown as mean ± standard error (SE). **P < 0.01. Lower panel: immunohistochemistry studies were carried out on frontal cortex sections from six autistic subjects and six age-matched controls using an anti-Wnt antibody (dilution 1:100). Weaker immunostaining of Wnt protein (dark brown color as indicated by arrows) was present in the autistic subjects compared with the controls (5**C**). Immunostaining density was quantified using Image J analysis (5**D**). Data are shown as mean ± standard error (SE). *P < 0.05. Scale bar: 20 μm.

## Discussion

Previously, a number of studies have suggested that abnormal functioning of glia and astrocytes may play a role in the development of autism. GFAP expression, a marker for astrocytes, has been reported to be significantly elevated in the cortex and cerebrospinal fluid of autistic subjects [13,14]. Other astrocyte markers such as aquaporin 4 and connexin 43 have also been shown to be altered in the brains of autistic individuals [20]. In particular, several recent studies have demonstrated that the abnormal functions of glia may also contribute to the progression of RTT, an X- linked autism spectrum disorder, and to the fragile X syndrome [15-18]. However, to date the information about glia/astrocyte development and function in the autistic brain is very limited. In this study, by employing western blotting and immunohistochemical approaches, we found that the morphology of astrocytes in the frontal cortex of autistic subjects was markedly altered compared with controls. The astrocytes in the autistic cortex exhibited significantly reduced branching processes, and the total branch length as well as the cell body size were significantly decreased. Further, the number of astrocytes was markedly increased compared with the controls. These results indicate that there is an astrocytosis in the autistic brain, and the structures of the astrocytes are altered.

RETRACTED

Astrocytes are the most abundant cells in the CNS and have been suggested to detect neuronal activity and modulate neuronal networks. Thus their structural integrity and sustained function are essential for neuronal viability [21-23]. The astrocyte branching processes are important structures, which can interdigitate between and closely approximate adjacent neuronal elements, thereby facilitating the local homeostasis of a range of molecules, including glutamate [24-26]. Studies have shown that the neurons depend upon the physical proximity of the astrocyte processes for normal function [23]. Torres-Platas *et al*. also reported that changes in astrocyte structures including branching processes, and cell body sizes may be significantly involved in mood disorders [27]. Thus, we suggest that the interruption of the astrocyte structures in the autistic cortex could critically impair neuronal function and the homeostasis of certain molecules such as glutamate, which may lead to the development of autistic-like behaviors.

Recently, studies have also shown that astrocytes have a complex, dual role in the local regulation of immune reactivity. They form the glia limitans around blood vessels restricting the access of immune cells to the CNS parenchyma [28]. Astrocytes have also been shown to be important regulators of neuroinflammation. Previous studies have demonstrated that astrocytes carry a series of germline-encoded pattern-recognition receptors (PRRs), which are important for the primary recognition of infectious agents [29]. Several cytokines, including IL-1 and IL-6, have been implicated in the induction and modulation of reactive astrogliosis and pathological inflammatory responses [30-34]. In addition, astrocytes have been reported to secrete inflammatory cytokine IL-6 [35]. Recently, various studies have suggested that abnormal immunity and localized inflammation of the central nervous system may contribute to the pathogenesis of autism. A number of studies including ours have demonstrated that cytokines including IL-6, IL-1β TNF-α and IFN-γ are elevated in the serum and brain tissue of autistic individuals [35-41]. We reckon that the astrocytic changes could result from an inflammatory process.

It will be important to determine whether the observed changes in astrocyte structure, as well as the astrocytosis found in the autistic brain are associated with elevated inflammatory cytokines such as IL-6. In this study, we did not determine the IL6 concentration in the same sample used for examining the astrocytes. Further studies can be conducted to examine cytokines including IL-6 and astrocytes in the same brain region at the same time. We suggest that it is also possible that the increased cytokines, in particular IL-6 in the autistic brain, could result from the astrocytosis.

RETRACTED

We next undertook to determine whether the alterations in the structure and density of astrocytes in the autistic brain also occurred in murine models of autism, including *NL3* knockdown mice and BTBR mice. We found that the morphology of astrocytes in the *NL3* knockdown mouse exhibited similar changes to that found in the autistic brain. They exhibit significantly reduced branching processes and total branch lengths, and as well the astrocytic cell body sizes were significantly decreased in comparison with the controls. Neuroligins are cell adhesion molecules localized postsynaptically in glutamatergic synapses, and interact with presynaptic neurexins to form heterophilic complexes, which likely play critical roles in synaptic transmission and differentiation of synaptic contacts [42-45]. A role of neuroligins in autism was implied by the discovery of deletions at Xp22.1 containing the *NL4X* gene in three female autistic individuals and a missense mutation (R451C) in *NL3* in two Swedish families with autism [46,47]. *NL3* knockdown mice have been shown to mimic certain human autistic behaviors [5]. Recent studies have demonstrated that *NL3* is expressed in many types of glia during the development of the nervous system. In particular, NL3 is expressed in the olfactory ensheathing glia, retinal astrocytes, Schwann cells, and spinal cord astrocytes in the developing embryo [48]. The *NL3* knock-down mouse in the current study was shown to exhibit autistic-like behaviors including increased anxiety, impaired cognition, vocal communication deficits and decreased social interactions (unpublished data). Thus, there is a possibility that alteration in astrocyte structure could be partially responsible for the development of autistic-like behavior in NL-3 knockdown mice. The mechanisms through which structural change in astrocytes could lead to behavioral changes remains to be further investigated. A limitation of this study was that we only had one *NL3* knockdown mouse that could be analyzed. More studies are needed to further confirm our observations.

We did not detect a significant change in the morphology of astrocytes in either the cortex or cerebellum of the BTBR mice, another murine model of autism. There were no significant differences in the number of astrocyte branching processes, the total length of processes orcell body size between the BTBR and control B6 mice. Nor did we find that there was an astrocytosis in the brain of BTBR mice similar to that found in the autistic brain. The density of astrocytes remained unchanged compared with the control mouse. However, we have not examined the orientation of the glial fibers. Recently, it was reported that there is a misorientation of selected glial fibers present in the BTBR forebrain [49]. This study found that the astrocytic processes were oriented dorsoventrally rather than mediolaterally in the cingulum and alveus at the levels of the striatum and hippocampus. The misorientation of glial processes was only found in brain regions that normally receive corpus callosal innervations, indicating that these findings are likely to be a consequence of callosal agenesis [49]. We therefore reason that although there are no changes observed in the astrocyte density, as well as in the number of branching processes and cell body sizes in BTBR mice, a misorientation of glial processes could lead to impairments in the functions of astrocytes, and consequentially impair synaptic plasticity and various neural functions and might contribute to the development of autistic-like behaviors. It has been demonstrated that astrocyte secreted proteins selectively increase hippocampal GABAergic axon length, branching, and synaptogenesis [50]. Whether the change in astrocytes in autistic subjects, or *NL3* knockdown and BTBR mice could impair the development of GABAergic axons, remains to be further studied.

RETRACTED

Both *NL3* knockdown and BTBR mice have been demonstrated to exhibit core autistic-like behaviors. Alterations found in the astrocytes of autistic subjects and the mice models imply that *NL3* knockdown mice and BTBR mice could offer opportunities for conducting biological studies to understand the mechanisms responsible for autism.

More and more evidence suggests that astrocytes are intimately associated with synapses and govern key steps in synapse formation and plasticity. However, we understand little about the molecular underpinnings of astrocyte development. It is unclear how astrocytes are specified at the appropriate developmental time from NPCs and how their development and maturation are regulated. The Wnt/β-catenin signaling pathway has been intensely studied as a key regulator of cell proliferation and cell fate during development, including neural development [10,23,51-53]. Recently, several studies have reported a role of Wnt/β-catenin signaling in the development of astrocytes [12]. It has been shown that Wnt/β-catenin pathway signaling regulates post-traumatic gliogenesis. Wnt/β-catenin pathway has also been demonstrated to act as a candidate regulatory circuit that controls mesencephalic dopaminergic neuron-astrocyte crosstalk [11]. In this study, we found that both Wnt and β-catenin protein expression were decreased in the brains of autistic subjects, suggesting that Wnt/β-catenin signaling activities are down-regulated. There is some evidence for a direct genetic link between Wnt2 and autism spectrum disorders. Two studies have found correlations between mutations of the *WNT2* locus and the incidence of autism in different populations [54,55]. Wnt2 has also been found to be expressed at lower levels in a mouse model of fragile X syndrome, a human disease strongly associated with autism [56]. Our findings imply that the decreased expression of Wnt and β-catenin may be associated with changes in astrocytes in the frontal cortex of autistic subjects. Further studies will be carried out to determine whether down-regulation of Wnt/β-catenin impairs the structure and density of astrocytes.

RETRACTED

## Conclusion

In summary, our study demonstrated that the morphology of astrocytes in the frontal cortex of autistic subjects was significantly altered compared with age- and sex-matched controls. The astrocytes in autisitc subjects exhibited significantly reduced branching processes, reduced total branching lengths and decreased cell body sizes. In addition, we detected astrocytosis present in the frontal cortex of autistic subjects. However these alterations of astrocytes are not detected in the autistic cerebellum. Interestingly, we found that astrocytes in the frontal cortex of the *NL3* knockdown mouse also showed significantly reduced branching processes, reduced total branching length and decreased cell body sizes, which mimic the changes in the autistic brain. These findings imply that the defects in astrocytes could impair neuronal plasticity and functions, and may partially contribute to the development of autistic-like behaviors in both humans and mice. We did not detect significant alterations in the density and morphology of astrocytes from the frontal cortex or cerebellum of BTBR mice. Recently, one study reported that there is a misorientation of selected glial fibers present in the BTBR forebrain. We suggest that even small changes like misorientation of glial fibers could affect astrocyte functions and consequently neuronal networks and lead to behavioral changes. Finally, we found that both Wnt and β-catenin protein expression was decreased in the brains of autistic subjects, which suggests that the Wnt/β-catenin signaling activities may be down-regulated. We suggest that the alteration of the Wnt/β-catenin pathway in the frontal cortex of autistic subjects could be one of the underlying mechanisms responsible for the observed changes of astrocytes. Our findings indicate that astrocytes may play an important role in the development of autism and may further suggest new potential therapeutic targets and strategies for intervention in autism.

RETRACTED

## Abbreviations

CNS: central neural system;GFAP: glial fibrillary acidic protein;HRP: horse radish peroxidase;MeCP2: methyl-CpG-binding protein 2;NPC: neural progenitor cell;PCR: polymerase chain reaction;PRR: pattern-recognition receptor;PVDF: polyvinylidenedifluoride;RTT: Rett syndrome;SE: standard error

## Competing interests

The authors declare that they have no competing interests.

## Authors’ contributions

AS, GW, FC, AY, ZT, AN, MS, FS, GM participated in data collection; LX, MM, WTB designed the study, secured the research funding and wrote the manuscript. All authors have read and approved the final manuscript.
